The article "Optimization of the Music Teaching Management System Based on Emotion Recognition" was published in 2022. Journal: Comput Intell Neurosci.

# Optimization of the Music Teaching Management System Based on Emotion Recognition

**DOI:** 10.1155/2022/4568041

**Published:** 2022-05-09

**Authors:** Yin Wang

**Affiliations:** Department of Public Arts, Henan College of Transportation, ZhengZhou 450000, China

## Abstract

Along with the development of social informatization, computer has been widely used in daily teaching and the technical support teaching management system, which can greatly improve the quality of students and teachers' information sharing and teaching, and is an important part of college information construction. Teachers' personal information, teaching information query, teaching file management, students' attendance, students' results query, teachers' evaluation, and so on constitute the music teaching information management system. Based on the Internet of things technology and emotion recognition, this paper mainly describes the design idea of the music teaching management system software, function design, and implementation scheme. The realization process of each subfunction module and hardware and software of the system is described in detail. In view of the characteristics of music teaching management itself, combined with the actual situation of music teaching, to form the system structure analysis, database design and data exchange, and other aspects of exploration, in order to establish a practical music teaching management system.

## 1. Introduction

At present, with the penetration of the concept of all-round education, the development of music education and teaching management has entered a new stage. Effective music education teaching management is the guarantee to improve the quality of music teaching [1–3]. How to reform and perfect the teaching management mode has always been an research and exploration direction. The credit system teaching management mode music art college, to realize the good interaction of teaching service, teaching management, and teaching research, training the compound talents needed by the society, has a very important role [4]. However, the traditional music teaching evaluation system is easy to fall into local extremes and slow convergence speed [5]. There have been few studies to fuse and expand the zero-crossing rate detection result to judge whether a piece of speech is a valid musical speech [6]. In this regard, we should constantly improve the system through in-depth research and give full play to the role of music education and teaching management mode. This is an important topic for music education in colleges and universities and also a new field of teaching management theory research [7].

With the ongoing reform of education, music teaching has become an important part of quality education. In music teaching process, the need to mobilize students' learning, abandon the boring and monotonous teaching mode and teaching content and make the students learn in a relaxed and pleasant environment music knowledge and skill in music [8]. The information assisted teaching of music education belongs to one part of educational information. Current development can provide a comprehensive support for the teaching process, such as registered in teaching, letting students pass the teaching evaluation, etc., which has been widely used in the university to teach computer-aided teaching software for assisted instruction. In the middle school education system, since the teacher computer level is not high, more computer assisted instruction is required to help teachers to reduce heavy work, improve teaching efficiency, but in fact, the computer-aided instruction system suitable for middle school education is very short [9–11].

The development of mobile Internet technology has a profound impact on people's learning mode. Now, mobile payment, WeChat, mobile phone QQ, and other applications have been closely related to life and work. The music teaching system based on Android makes full use of the existing mobile Internet technology and network technology to build the foundation set information management student music work music practice management [12]. Online classroom management information to inform management in a body's comprehensive teaching platform to provide professional support for professional music teaching and learning, for distance learners by a mobile phone network provides a great convenience, mainly reflecting in teaching and learning can provide recipients with learning contents, learning process, and learning methods [13]. This diversified learning mode not only meets normal classroom learning but also enables learners to complete exercises or tests through the platform, so as to achieve better learning effects. The online teaching and learning platform based on the Android platform makes the current hottest mobile Internet better, reflecting the advantages of completing learning tasks through mobile phones at anytime and anywhere [14]. Moreover, the portable platform can make full use of learners' scattered time to complete learning and practice, ensuring the learning effect and systematic charging. In addition, music teaching has strong professional characteristics, such as the need to identify sound through notes, etc., and the system makes full use of Android platform media technology, providing a concise interface design to complete the music professional teaching system [15, 16].

Thesis design study of the music teaching system that can be used in the teaching of the music lets learners through class often learn operation practice and implements comprehensive information notification function of the music learning platform, makes learning in the music learning environment, which has changed the past model that online learning is just practice and increases the learning effect [17]. This system can be applied to other professional learning systems; the functional model of the teaching learning system dynamic model can be applied and popularized, the students' learning mode practice mode can be adopted in the same online learning system, improving the learning interest of learners and increasing the learning effect. The rich classroom teaching content music classroom teaching assistant system will effectively change the traditional music classroom's old teacher to teach students to listen to the teaching mode music classroom teaching assistant system, which can provide a variety of bathhouse teaching scenes, such as playing the piano to make up music to appreciate music; it can also provide classroom tests, such as rhythm training. At present, the proportion of students who can effectively use computers and the Internet to study is quite high [20].

As shown in Figure 1, the frequency response of the filter in IoT is given, which may affect the emotion recognition. Its essence is a school education computer tool used in the school education management system as a whole and helps teachers to carry out information planning for teaching resources, which can reduce the workload of teachers and improve the quality of teaching effectively. Of course, music teaching information management is not only the application of computer but also gives full play to the potential of teachers and students' quality education intelligence, with reference to its management system, in-depth mining, and development. With the specific characteristics of music teaching to design, it will eventually form a virtual music teaching information management system co-existing with the development of school teaching management and mutual use. In fact, in the past, many schools have developed related auxiliary systems, but in the music assisted teaching, because of its large workload, different situations are complex and cannot form a more standardized and general management system. Thus, it is urgent to realize the scientific system and distribution of information management.

The main features include the following: expanding the beneficiary groups. When the information of music teaching resources spreads rapidly on the network, students can obtain music teaching resources, so learning will not be affected by region and time. In this context, more and more students will enjoy the convenience brought by teaching information. Promoting students' autonomous learning. With the help of music teaching assistant system, students can choose the learning time, place, and content according to their own situation. Autonomous learning ability will be quickly improved, learning efficiency can also be greatly improved. This paper introduces the research background and status of the university music education teaching management system and analyzes the deficiencies of the university music education teaching management research status. In the overall demand analysis of the system, the use case analysis of the module is carried out through the overall business overview, and the use case description. In addition, the college music education's nonfunctional requirements were analyzed, and the teaching management system in colleges and universities music education teaching management system, based on the analysis of the overall demand for architecture choice, puts forward the target system architecture technology architecture, the system architecture design, architecture framework on a detailed module design and database design. Through the relationship between core business classes and core business objects, each module is described and analyzed in the form of a sequence diagram to complete the realization process of college music education and the teaching management system. The key technologies and common methods used in the realization are described, and the key modules involved in the system are also displayed. In addition, the university music education teaching management system is systematically tested through test cases.

The main contributions of this paper can be concluded as follows:

1. The main problems of the current music teaching management system are as follows: poor teaching effect, easy to appear in the management of loopholes, and subjective interference.
2. This paper designs an English teaching management system based on the Internet of Things technology and emotion recognition, which not only has good operability but can also carry out teaching management automatically.
3. Based on the above framework, we also combined with the teaching situation of time to optimize the proposed method, in order to obtain better management effects.

## 2. Related Work

After 1990, Internet technology and multimedia technology received rapid development, teaching resources, and communication for education, etc., due to the support of the Internet, produced earth-shaking changes, and is no longer the traditional intelligent teaching system (ITS); now, students can choose their favorite teachers, what they want to learn the course, anytime and anywhere according to their own time, their own characteristics, according to their favorite way of learning, through the Internet in the world's educational resources. Compared with the domestic research on the intelligent education system, there are more foreign studies in the 1980s. The research of ITS is influenced by the development of cognitive theory and teaching theory, which is reflected in that the intelligent teaching system GUIDON (combined with MYCIN), which developed an important milestone in the development of ITS. For the understanding of the intelligent teaching system, different scholars have different understandings. The purpose of the research teaching system is to realize the intelligentization of human cognitive teaching and learning by means of computer and network technology, which can improve the efficiency of students' learning and reduce the workload of teachers. In the United States and Europe, English teaching management systems are also gaining attention.

The education information resources can be shared in a short time, which can greatly improve the efficiency of teaching and learning. The high-speed development of the Internet provides convenience for this. The network teaching management information system is an important part of education informatization and also the foundation of education informatization. The principle is very simple: it is to combine the intelligent artificial technology of computer with the management method and information organization in hypermedia to create an intelligent information processing technology. In this teaching method, the explanation can be brought to students through hypermedia, including text rich multimedia content including sound and images. Moreover, this module can control (adaptability) the use of reasoning technology to show the teaching strategy and teaching content, through this way for students to guide the target. At present, the development this new teaching system has become the core frontier content of scientific research in the applied field of computer network teaching. By contrast, how far has China's English teaching management system developed?

In recent years, China has been continuously promoting educational reform, involving fields including educational informatization (universities), multimedia teaching (primary and secondary schools), and quality education. According to the relevant investigation of the education department, as of 2005, developed eastern region of the multimedia teaching has been very popular, many schools have already completed the closed-circuit television (CCTV) and the construction of campus network. According to statistics, every school an average of two networks in the classroom. Two phonetic teaching rooms and three multimedia classrooms of primary and secondary schools are on the campus network and CCTV integration and implementation. The multimedia network technology is applied in the teaching process to realize the unified management and optimization of education, teaching and teaching resources, so that the teaching effect is more obvious. At the same time, in view of the part of the teachers are not good at using multimedia teaching, many middle and primary schools are opened for education workers' training After a period of training, many teachers now have mastered operating the computer or are capable of using a computer to make the multimedia teaching tools to write. Nearly, half of the teachers can use computers to make teaching web pages and courseware, and gradually in the teaching process to use higher teacher strength of part of the school also for part of the curriculum, completed the development of teaching assistance platform, for the teacher's work has high value.

Some education and training institutions set up charge for the online learning system, by buying learning resources, the payment method to complete the pay resources can be unlimited learning, the learning mode to a certain extent, becomes a useful supplement school garden education, let more did not have a chance to go to school for learners to obtain professional knowledge, accepted the professional training. These online learning systems are generally based on courseware playback, emphasis on knowledge acquisition, but lack of corresponding exercises. General learners can complete learning tasks by registering online accounts and ordering learning resources online. The characteristics of music professional listening for training. Those who learn the basics of music for the general public; their appearance effectively solved the difficult to traditional music teaching to solve the problem. Send some music teaching software are different, each have short, applicable to surface also each are not identical. In the process of music teaching, we should choose appropriate music teaching software to assist the teaching according to the actual situation. To make full use of these software, we should first understand the characteristics of this software.

As China strives to become a big manufacturing country, the manufacturing industry needs more and more high-quality skilled talents. The report, the party's 18 to speed up the development of modern vocational education, strengthen professional skill training, raise the labor employment entrepreneurship ability of higher vocational education in the development of industrial structure adjustment of economic and social transformation not replaceable important role, vigorously develop China's higher vocational education is imminent, the trend of the system enterprises needs to be of more highly qualified graduates in higher vocational colleges, and how to embody high quality, many higher vocational colleges to music education in the first place; our hospital is not exceptional also, music education has affected more and more students, so the difficulty of music teaching management is getting bigger and bigger. How to reduce the difficulty of music education management? First of all, we can use the advantages of computer and Internet to design a set of music education management software which can be efficient and reflect the high quality of higher vocational education.

After entering the 21st century, with the desktop computer office automation, the investment in quality-oriented education in university education funds gradually increased; each university developed and purchased the corresponding combined with the actual course management system online course design and teaching data management system, but in some aspects to be improved, the performance is as follows: The library has purchased a large number of literature resources and teaching materials. For class again most of no use, the learning school and no professional quality information data, such as teaching plans and question bank, let the teachers teach free search and compiling system, no unified standard service teaching, not timely organization of teacher professional development based on the relevant teaching of the college information repository (2) the music teaching management software is rarely at home, a lot of a lot of management software, and with the music teaching management software is very few, even some famous music professional schools are few music teaching information management software (3) teaching resource update teaching includes not only the use of teachers resources not in time but also use of resources, including students and teaching. No doubt these resources are very valuable. If online courses can be designed, interactive online course education can save some rare materials in the class.

## 3. Optimization of the Music Teaching Management System by IoT and Emotion Recognition

### 3.1. Flowchart of the Optimization Method

Through three-step coding, this paper clarifies the psychological factors, social demands, internal operation, external environment, sociology, demographic variables of the performance of music teaching management system, and combs out the relationship structure between the main categories. Based on this combined with Internet technology and emotion recognition method, a large-scale music teaching management system is constructed. The whole system of the method is given in Figure 2.

According to the model of music teaching management system, this paper proposes the following four types of hypothesis to carry out research: (1) the influence of individual students' classroom behavior on the teaching system; (2) hypotheses about the correlation between situational factors and academic classroom behavior; (3) the moderating effect hypothesis of dual-channel mental accounts; and (4) hypothesis of the influence of student number changes on the teaching system.

### 3.2. Internet of Things System

In this paper, frequency domain technology is used to optimize the teaching management system. Before subsequent processing, the original signal is filtered according to the following formula:

(1) $$\begin{array}{c} H\left(z\right)=2-\alpha z^{-1},\\ E_{G}^{N}=\text{yz}\left(s-b\right)+\left(1-y\right)z\left(-b-k\right)+\left(1-y\right)\left(1-z\right)\left(-b\right). \end{array}$$

So, the function expression for the case is as follows:

(2) $$\begin{array}{c} w\left(n\right)=\left\{\begin{array}{cc} 0, & 0<n<N-1,\\ 1, & n\geq 1\text{ or }n\geq N+1. \end{array}\right) \end{array}$$

Then, the other is the function equation based on the following cosine window:

(3) $$\begin{array}{c} w\left(n\right)=\left\{\begin{array}{cc} \left(1+\alpha \right)+\alpha \;\sin\left|\frac{2\pi n}{N}\right|, & 0\leq n\leq N,\\ 1, & n=\text{else.} \end{array}\right) \end{array}$$

The specific function expression of the cosine window is shown below:

(4) $$\begin{array}{c} w\left(n\right)=0.5\left[\left(1+\alpha \right)+\alpha \;\sin\left|\frac{2\pi n}{N}\right|\right]R_{N}\left(n\right). \end{array}$$

The expected revenue of sports venues choosing not to reduce or exempt tickets or not to issue sports consumption vouchers is as follows:

(5) $$\begin{array}{c} E_{S}^{N}=xz\left(b-p\right)+\left(1-x\right)zb+\left(1-x\right)\left(1-z\right)b. \end{array}$$

Then, the rough estimation of spectral feature correlation can be further obtained as follows:

(6) $$\begin{array}{c} E\left(S\right)=yE_{S}^{Y}+\left(1-y\right)E_{S}^{N}. \end{array}$$

which can be transferred into the following:

(7) $$\begin{array}{c} Z_{n}=\sum_{m=0}^{+\infty }\left|\mathrm{sgn}\left[x\left(m\right)\right]+\mathrm{sgn}\left[x\left(m\right)-1\right]\right|w\left(n+m\right). \end{array}$$

Then, the average energy of the sign at a certain moment is as follows:

(8) $$\begin{array}{c} E_{n}=\sum_{m=0}^{+\infty }{\left|x\left(m\right)\cdot w\left(n+m\right)\right|}^{2}w\left(n+m\right). \end{array}$$

Then, the update gate can be expressed as follows:

(9) $$\begin{array}{c} z_{t}=\sigma \left(W^{z}x_{t}+U^{z}h_{t-1}\right), \end{array}$$

After that, the reset gate *r*_*t*_ is given as shown below:

(10) $$\begin{array}{c} r_{t}=\sigma \left(W^{r}x_{t-1}+U^{r}h_{t+1}\right),\\ C\left(n\right)=\sum_{m=0}^{N-1}\frac{S\left(m\right)\cos\left(\pi \text{ nm}+0.5\pi n\right)}{2}. \end{array}$$

## 4. Experimental Results and Analysis

### 4.1. Introduction to Experimental Data Set

Through system analysis and system outline design, the function of the system has a detailed understanding, a system is supported by the database, so it is necessary to complete the design of the system database, in this part by the system database conceptual model and physical structure design to describe the design of the system database.

As we know, database design includes three major parts: (1) to use the database conceptual model diagram to describe the conceptual design and logical design of the system, (2) to describe the core table structure of the physical design of the database table design is a part of the database physical design, and (3) through the description of the data table structure to achieve the physical design of the database select part of the table in this part, to describe its physical structure. In conclusion, the characteristics of the data set selected in this paper are consistent with the method proposed in this paper, so it can be the validation platform of the method.

### 4.2. Experimental Results Analysis

As shown in Figure 3 when music teachers think a teaching repertoire has a special significance, or to a repertoire of teaching methods of teaching, Have their own unique indirectly when can share to the colleagues around, let the other music teachers discuss the piece has a variety of teaching methods to share way, one is through sharing tools to share to the specified teacher, accept share the teaching material teachers can see what is shared; It is shared to the group designated by the music teacher, and the teachers in the group can see the shared material; Third, share to friends and make them see the shared content.

In the class design, resources is an entity class, which is used for the maintenance of music jobs. Resources ID is a resource number, file is a resource file object, and Resources File is a resource file class, which is used to realize the upload check of resource file display and delete operations, which are implemented by controlling classes show file and upload. The following describes the process of uploading a resource file as an example.  Figure 4 shows the sequence of uploading a resource file.

In Figure 4, the user first invokes the resource to check the details of the music through the user interface, then uploads the file through the resource, and checks the file through the method of the resource file (mainly to check whether the file format is supported). After the check passes, upload the resource file to the upload class. Music practice is done through mobile phones. The practice questions reflect the practice effect through the sound of mobile phone, including accompaniment practice, test questions practice and masterpieces practice. Therefore, the management module of students' scores is designed, and it has the function of importing scores of different classes.

Figure 5 gives the F-measure rate of systematic reviews. The website is mainly composed of resource center problem consultation forum teaching assistance and background management, and the specific functions are as follows: Resource center: teachers can upload, download, and delete resources. Students can choose teachers to consult for online consulting management. Teachers can answer questions based on the data. Users' personal home page: the user interface is designed to teach music teachers according to their own needs to set their own personal database, save the teacher in class requires some teaching materials (audio staff chords lesson plans) with now is to find time. According to most music teachers' teaching habits, the teacher user's personal homepage as common repertoire and course materials. The index under this classification and the teaching materials under the index can be compiled before the start of classes in each semester. Because the content of music textbooks is fine-tuned each year, the content of course materials does not change much.

Figure 6 shown the relationship between series value and the number of experiments. It can be seen from the figure that different series of music types have different responses to time and do not show the regularity of their characteristics.

Along with the computer application development process continuously improve, for detecting program correctness full colorful safe sex software testing methods, such as more and more rich, more and more systems. Thus, the developers can choose the application of sequence of different application testing methods of the digital music classroom teaching assistant system according to the application scope of music. Compared with other aspects, classroom teaching pays more attention to the accuracy of each function of the system. The test method adopts is mainly black box test, which is also called function test. It detects whether each function can be used normally through testing. As can be seen from Figure 7, the corresponding time and recognition time of different kinds of music are quite different.

In addition, the recognition time and file recording time of test and actual are given in Figure 8 where the red line represents the test and the black line represents the true value; it can be seen that different music have different impacts on the optimization of music teaching management system, and the difference is also large.

## 5. Conclusions

Music teaching process, through the teacher's summary is helpful for teachers to timely summarize the problems encountered in the teaching process, adjust teaching methods and teaching methods, improve teaching quality, and increase feedback. Auxiliary teaching in the form of multimedia can stimulate students' interest and improve their memory and understanding.

In the process of learning, students can search for key words in the fastest way to a satisfactory solution to a specific part of the research and testing, students can search or through the form of direct courseware data retrieval learning. At the same time, when students lack of learning purpose, they can timely consult the music teacher, who will guide students to learn. This thesis mainly focuses on the design and development of teaching assistance system. The design and optimization of music teaching management system based on Iot and emotion recognition is proposed, which is beneficial to software development and development schedule control and quality control.

## Figures and Tables

**Figure 1:** Enhanced filter frequency response.

**Figure 2:** Architecture of Internet of Things and music teaching assistant platform.

**Figure 3:** Sequence diagram of teaching track management module.

**Figure 4:** Resource file uploading sequence diagram.

**Figure 5:** System measures the F rate of different music.

**Figure 6:** Response time comparison.

**Figure 7:** Performance test data.

**Figure 8:** Recognition time and file recording time.

## Data Availability

The data used to support the findings of this study are available from the corresponding author upon request.
